# Verification of Ferroptosis Subcluster-Associated Genes Related to Osteosarcoma and Exploration of Immune Targeted Therapy

**DOI:** 10.1155/2022/9942014

**Published:** 2022-09-28

**Authors:** Mingyang Jiang, Yiji Jike, Fu Gan, Jia Li, Yang Hu, Mingjing Xie, Kaicheng Liu, Wentao Qin, Zhandong Bo

**Affiliations:** ^1^Department of Bone and Joint Surgery, The First Affiliated Hospital of Guangxi Medical University, Nanning, China; ^2^Department of Urology Surgery, The Affiliated Hospital of Youjiang Medical University for Nationalities, Baise, China; ^3^Department of Pathology, The First Affiliated Hospital of Guangxi Medical University, Nanning, China

## Abstract

**Background:**

Despite tremendous advances in treating osteosarcoma (OS), the survival rates of patients have failed to improve dramatically over the past decades. Ferroptosis, a newly discovered iron-dependent type of regulated cell death, is implicated in tumors, and its features in OS remain unascertained. We designed to determine the involvement of ferroptosis subcluster-related modular genes in OS progression and prognosis.

**Methods:**

The OS-related datasets retrieved from GEO and TARGET database were clustered for identifying molecular subclusters with different ferroptosis-related genes (FRGs) expression patterns. Weighted gene coexpression network analysis (WGCNA) was applied to identify modular genes from FRG subclusters. The least absolute shrinkage and selection operator (LASSO) algorithm and multivariable Cox regression analysis were adopted to develop the prognostic model. Potential mechanisms of development and prognosis in OS were explored by gene ontology (GO), Kyoto Encyclopedia of Genes and Genomes (KEGG), and gene set enrichment analysis (GSEA). Then, a comprehensive analysis was conducted for immune checkpoint markers and assessment of predictive power to drug response. The protein expression levels of the three ferroptosis subcluster-related modular genes were verified by immunohistochemistry.

**Results:**

Two independent subclusters presenting diverse expression profiles of FRGs were obtained, with significantly different survival states. Ferroptosis subcluster-related modular genes were screened with WGCNA, and the GESA results showed that ferroptosis subcluster-related modular genes could affect the cellular energy metabolism, thus influencing the development and prognosis of osteosarcoma. A prognostic model was established by incorporating three ferroptosis subcluster-related modular genes (*LRRC1*, *ACO2*, and *CTNNBIP1*) and a nomogram by integrating clinical features, and they were evaluated for the predictive power on OS prognosis. The 20 immune checkpoint-related genes confirmed the insensitivity to tumor immunotherapy in high-risk patients. IC50s of Axitinib and Cytarabine suggested a higher sensitivity to the targeted drug. Finally, the quantitative reverse transcription-polymerase chain reaction (qRT-PCR) and immunohistochemistry were consistent with bioinformatics analysis.

**Conclusion:**

Ferroptosis are closely associated with the OS prognosis. The risk-scoring model incorporating three ferroptosis subcluster-related modular genes has shown outstanding advantages in predicting patient prognosis.

## 1. Introduction

Osteosarcoma (OS), a prevalent primary malignancy in the bones of teenagers [1], is most often located in the long bone epiphysis, especially around the distal femur or proximal tibia of the knee joint. OS features an extraordinary incidence of disablement and a poor prognosis, primarily because of its susceptibility to metastases (particularly to the lungs) [2]. Current clinical characteristics such as metastasis in OS patients remain crucial for risk stratification and treatment strategy selection. However, individuals possessing the same clinical features and treatment show different clinical outcomes [3]. This phenomenon may be due to the genomic complexity and instability in OS [4]. Therefore, optimizing the prognostic prediction of OS from a molecular genetics perspective may provide more accurate risk stratification and the development of personalized treatment strategies for OS patients.

In previous studies, several prognostic models for OS have been developed. The prediction model developed using 5 metastasis-associated genes displayed a good evaluation power for the prognosis of OS patients [5]. The prognosis prediction model for OS patients based on 14 autophagy-related genes showed promising efficacy for survival prediction in OS patients [6]. A prognostic model consisting of 21 immune-associated genes also showed accurate ability for the overall survival prediction of OS patients [7]. Recently, a prognostic model, established by Lei et al. based on 12 ferroptosis-related genes (FRGs), showed a well predictive efficiency, and researchers demonstrated the influence of FRGs on the tumor-immune microenvironment [8].

Ferroptosis is iron-dependent, having a fatal lipid peroxidation accumulation with tumorigenesis and therapeutic response in various tumors [9]. Ferroptosis displays unique characteristics different from apoptosis, regulates cancer cell proliferation, and has shown potential value in tumor research [10]. The main mechanisms of ferroptosis involve ROS generation. Intracellular ROS content is tightly related to tumorigenesis, angiogenesis, metastasis, and invasion of tumor tissue [11]. Combined view, exploring the clinical value and underlying molecular mechanisms of ferroptosis in OS is essential.

In the present research, we designed to develop a risk-scoring model to quantify the expression level of ferroptosis subcluster-related modular genes in OS and explore its prognostic and targeted therapeutic role.

## 2. Materials and Methods

### 2.1. Data Sources

As a training set for this study, the GSE21257 dataset, consisting of mRNA sequencing data of 53 OS patients and clinical information material, was sourced from the Gene Expression Omnibus (GEO) database (https://www.ncbi.nlm.nih.gov/geo/). The testing set was sourced from the Therapeutically Applicable Research to Generate Effective Treatments (TARGET) database (https://ocg.cancer.gov/programs/target), including 85 samples (TARGET-OS). The Ferroptosis Database (FerrDb, http://www.zhounan.org/ferrdb/) was utilized for selecting FRGs.

### 2.2. Identification of Molecular Subclusters of FRGs in OS

The “limma” package was used for intergroup difference analysis of each subtype, and the calibrated *P* value less than 0.05 and the absolute value of the logarithm of the multiple of difference (|logFC|) greater than or equal to 1 were taken as the inclusion criteria of the differential genes [12]. The obtained differentially expressed genes (DEGs) were included in the TARGET osteosarcoma data set for consistent clustering analysis using “ConsensusClusterPlus” packages, and the proportion parameter of the resampled samples was 80%. The maximum evaluated number of categories was 9, and the clustering distance was selected as “Euclidean”. The optimal *K* value of the number of clusters was selected and divided into different subclusters according to the *K* value.

### 2.3. Identification of Related Genes among Different Molecular Subclusters

The coexpression network between genes and clinical traits was constructed with the R package “WGCNA” [13], and samples with an expression less than 0.5 were removed. Then the scale-free distribution topology matrix was computed. The “pickSoftThreshold” function was applied to select the best soft threshold *β*, with the Pearson correlation coefficient calculated. The neighbor-joining matrix constructed with the weighted correlation coefficient was transformed into a topological overlap matrix to construct a clustering tree. The module including greater than 150 genes was retained, and the modules with similarities greater than 0.25 were merged. Finally, the genes in the module related to the FRG molecular subclusters were extracted.

### 2.4. Construction and Verification for the Prognosis Model Based upon Differential Molecular Subclusters-Associated Genes

The TARGET-OS dataset was used as the testing set. The univariate Cox regression analysis of the training set was conducted for genes related to OS prognosis from the GSE21257 dataset using the R package “survival”. Then genetic analyses were implemented using the least absolute shrinkage and selection operator (LASSO) regression method via the “glmnet” package. *λ* min of the lowest error was opted after 10-fold cross-validation [14] for constructing a stable prognosis model. Multivariable Cox regression analysis was then performed to develop the optimal model and calculate the regression coefficient and risk score as ∑_*x*=1_^*n*^(coef*x* × Expr*x*). The median was used as a criterion for grouping. The model efficacy determination generated the Kaplan-Meier (K-M) survival and receiver operating characteristic (ROC) curves. In addition, for more intuitive prediction, we incorporated age, gender, tumor location, and metastasis into the model, constructed a nomogram using the “Regplot” package in R, and validated the stability.

### 2.5. Functional Analysis and Mechanism Study of Ferroptosis Subcluster-Related Modular Genes

Functional enrichment analyses of Gene Ontology (GO) and Kyoto Encyclopedia of Genes and Genomes (KEGG) pathways were employed to characterize differential gene functions using the R package “clusterProfiler”, and the adjusted *P* < 0.05 items from enrichment results were displayed.

### 2.6. Gene Set Enrichment Analysis (GSEA)

GSEA analysis of high and low expression groups was performed using the GSEA function of the “clusterProfiler” package for the gene sets c2.cp.kegg.v7.4.symbols.gmt and c5.go.v7.4.symbols.gmt, and the first seven with *P* < 0.05 were selected for presentation. Gene sets were considered significantly enriched when *P* < 0.05, the normalized enrichment score (|NES|) exceeded 1, and the false discovery rate (FDR) adjusted *P* value was less than 0.25.

### 2.7. The Predictive Power of Target Drugs Response

The half-maximal inhibitory concentrations (IC50s) of target therapeutics were graphed with the “ggplot2” and “pRRophetic” packages in R, and box plots indicate the association of IC50s with the two risk groups.

### 2.8. Quantitative Reverse Transcription-Polymerase Chain Reaction (qRT-PCR) Analysis

Human osteosarcoma cells MG-63 and human osteoblast hFoB1 (Procell, China) were cultured following the protocols. When the confluence rate reached 70%~80%, cells in the logarithmic growth stage were taken for follow-up study [12].

RNA was extracted from each group of cells using the TRIzol kit (Invitrogen, USA). The RNA concentration was determined by NanoDrop2000 spectrophotometry (Thermo, Wilmington, USA). Reverse transcription was performed by the Qiagen QuantiTect Reverse Transcription Kit (Qiagen, Hilden, Germany), followed by Real-time qPCR conducted using SYBR-Green (Takara, Japan). The primers used in PCR were designed and synthesized by Shanghai Shenggong Bioengineering Co. PCR amplification was performed in 40 cycles by denaturing at 95°C for 15 s, annealing at 60°C for 30 s, and elongation at 60°C for 30 s. The gene expression was standardized with the GAPDH. Primer sequences are listed in Table 1. Data analysis adopted the 2-*ΔΔ*CT method.

### 2.9. Immunohistochemical Validation

Ten sarcoma and three paracancerous tissues of OS patients diagnosed by the First Affiliated Hospital of Guangxi Medical University were subjected to immunohistochemical examination. The tissue slices were deparaffinized with xylene, rehydrated, antigen-repaired with Tri-EDTA (pH = 9), incubated with H_2_O_2_, and blocked with sheep serum. Sections were incubated with primary antibodies (ACO2 [Cat number: 11134-1-AP; Rosemont, USA], LRRC1 [Cat number: 10128-2-AP; Rosemont, USA], and CTNNBIP1 [Cat number: bs-4095R; Rosemont, USA]) and sequently secondary antibodies. Diaminobenzidine coloration and hematoxylin staining were conducted. 10 random visual fields (×400) were observed by two researchers independently. The positive protein expression of diaminobenzidine was brownish yellow.

### 2.10. Statistical Analysis

R software (Ver. 3.6.2) was used for data analyses. The K-M survival curve was adopted for the relationship between the prognosis of each eigenvalue and the Log-rank test for evaluating survival curves. Independent prognostic factors, identified using Cox regression analysis of univariate and multivariate, were screened for overfitting using Lasso regression. Continuous variables (e.g., age) were transformed into dichotomous variables. The data comparison of the two groups was conducted through a two-tailed *t*-test and, when appropriate, Welch's *t*-test. *P* < 0.05 was considered statistically significant.

## 3. Results

### 3.1. Constructing FRG Molecular Subclusters

According to 61 FRGs of 53 OS samples from the GSE21257 dataset, 51 FRGs were identified as DEGs. The obtained DEGs were then included in the target osteosarcoma dataset for consistent clustering analysis using the “ConsensusClusterPlus” software package. Finally, two independent subclusters were obtained based on the principle of minimal crossover between cluster strata (Figures 1(a)–1(c)). Survival analysis of subclusters showed that the overall survival of cluster A was significantly outperformed by cluster B (Figure 1(d)).

### 3.2. The WGCNA Analysis Based on FRG Molecular Subclusters and the Construction of a Prognostic Model

In the WGCNA analysis, we calculated a soft threshold *β* = 6 using R software and then obtained a hierarchical clustering tree using the dynamic cutting method (Figure 2(a)). A total of 7 modules were obtained after merging similar modules. The Pearson correlation matrix of the module features showed that the “turquoise” and “blue” modules were correlated with the characteristics of different FRG molecular subclusters in OS (Figure 2(b)). The “turquoise” module containing 626 genes was more highly correlated (*R* = 0.63, *P* < 0.001) and was chosen for the following analysis. With *P* < 0.01 as the screening condition, 19 OS prognosis-related genes were obtained (Figure 2(c)). To prevent overfitting of the model, we took Lasso regression analysis to test these 19 genes and determined that there was no overfitting for these genes. The changes in the independent variables are shown in Figures 2(d) and 2(e). Finally, three prognostic markers were identified (Figure 2(f)), besides a risk-scoring model was developed. RiskScore = 0.7576∗ACO2 − 0.9240∗CTNNBIP1 + 1.3637∗LRRC1.

### 3.3. Validation of the Prognostic Model

The median risk score of the training set was adopted as a criterion for high and low-risk grouping, and survival analysis indicated a negative correlation of the risk score of OS patients to prognosis (Figures 3(a),and 3(b)). The high-risk group exhibited higher *LRRC1* and *ACO2*, and lower *CTNNBIP1* expression (Figure 3(c)). K-M curves in Figure 3(d) demonstrated significant survival differences between the two groups. The low-risk group had a significant survival advantage. In addition, ROC analysis showed that the area under the curve (AUC) at 1-, 3-, and 5-year survival were 0.918, 0.844, and 0.875, respectively (Figure 3(e)). It suggested a good predicted capability of the model. In addition, the prediction accuracy was assessed by calibration curves (Figure 3(f)). There was high agreement between actual and predicted 1-year, 3-year, and 5-year survival rates compared to the reference line.

To ensure the model's accuracy, we validated the established model on the external validation set (TARGET-OS). Intergroup survival analysis revealed a negative correlation between the risk score of OS patients and prognosis (Figures 4(a) and 4(b)). The heat map for the three genes in Figure 4(c) displayed the same change trend as the results in the training set. Moreover, K-M curves of the TARGET-OS dataset showed notable survival differences (Figure 4(d)). ROC analysis showed that the AUC at 1-, 3-, and 5-year survival were 0.844, 0.687, and 0.677, respectively (Figure 4(e)). Finally, the consistency between the actual and the predicted 1-year, 3-year, and 5-year was evaluated by calibration curves (Figure 4(f)), which suggested a good accuracy in internal and external validation datasets.

### 3.4. Correlation of Risk-Scoring Model to Clinical Features

In the constructed prediction model of risk based on three ferroptosis subcluster-related modular genes, we incorporated clinical characteristic values in OS, including age, gender, tumor location, and metastases. Then the analysis of eigenvalues was followed by the Cox regression analysis of univariate and multivariate and indicated the association between prognosis in OS, and metastases and risk score which were independent prognostic factors (Figures 5(a) and 5(b)). In Figure 5(c), the results showed differences in risk score between the subgroups of gender and metastases.

### 3.5. Establishment of the Nomogram

In Figure 6(a), a nomogram was plotted for survival prediction of OS patients by scoring each characteristic value. In addition, we used ROC curves to determine their accuracy (Figure 6(b)). This risk score corresponded to the highest AUC value (AUC = 0.917) compared to other clinical characteristics. Decision curve analysis (DCA) indicated a great potential for clinical utility (Figure 6(c)). It further demonstrated the clinical usefulness of the signature. The above data proved the model's capability of accurately predicting OS survival.

### 3.6. Functional Enrichment Analysis

626 genes from the “turquoise” module were analyzed by GO and KEGG functional enrichment with R package “clusterProfiler” (Figures 7(a)–7(d)). GO analysis revealed the enrichment of biological processes (BP) such as mRNA catabolic, RNA catabolic, translational initiation, and nuclear−transcribed mRNA catabolic as well as the enrichment of cellular constituents (CC) in focal adhesion, ribosome, and mitochondrial protein complex. KEGG enrichment analysis showed that they are associated with various metabolic pathways, such as protein processing in the endoplasmic reticulum, oxidative phosphorylation, nucleocytoplasmic transport, and citrate cycle (TCA cycle).

To identify the differences in function between different risk groups, GSEA was implemented. GO enrichment analysis showed significant enrichment of the low-risk group in adaptive immune response, granulocyte migration, humoral immune response, and immune response regulating signaling pathway (Figure 8(b)). KEGG enrichment analysis revealed a significant association of the high-risk group with the cell cycle, citrate cycle, steroid biosynthesis, and TGF-beta signaling pathway (Figure 8(c)), and a significant association of the low-risk group with the cytokine receptor interaction, the intestinal immune network for IgA production, chemokine signaling pathway, and toll-like receptor signaling pathway (Figure 8(d)).

### 3.7. The Risk-Scoring Model Was Associated with Immune Checkpoint Markers and Response to Targeted Therapy

For association analysis of model and immune checkpoint-related genes, 19 were low and 1 was highly expressed in the high-risk group (Figure 9(a)). According to predicted IC50s, the response to targeted drugs differed significantly between the two risk groups. For Axitinib and Cytarabine, IC50s were lower in the high-risk group, suggesting stronger sensitivity to the target drug (Figures 9(b) and 9(c)). In contrast, the high risk for Roscovitine is related to a lower sensitivity (Figure 9(d)).

### 3.8. qRT-PCR

The expression level of LRRC1 and ACO2 were notably higher in two osteosarcoma cells than in human osteoblasts. At the same time, the CNTTBIP1expression was not consistent between the two groups (Figure 10).

### 3.9. Immunohistochemical Validation

ACO2 and LRRC1 were significantly more expressed in osteosarcoma tissues than in paracancerous tissue, while CTNNBIP1 is the opposite (Figures 11(a)–11(f)).

## 4. Discussion

OS is a prevalent primary malignancy in the bones with high aggressiveness. Despite significant advances in treatment options such as surgery and chemotherapy, considerable patients still experience recurrence or metastasis [15]. When metastasis occurs, or response to initial therapy is poor, the 5-year survival rate reaches just 20% [16]. Thus, the exploration and characterization of novel prognosis biomarkers are vital for making appropriate clinical decisions and improving patient prognosis.

In the present work, two molecular subclusters were first determined according to the expression levels of 51 differentially expressed FRGs and demonstrated distinctly differing survival states. These two FRG molecules subcluster were identified using WGCNA to identify ferroptosis subcluster-related modular genes. Gene function enrichment analysis of this modular gene was performed. The results showed that ferroptosis subcluster-related modular genes could influence cellular energy metabolism. Energy metabolism is closely related to tumor progression. Indeed, tumor cells usually undergo energy metabolism reprogramming to meet the requirements for proliferation and survival in an unfavorable environment [17]. The tricarboxylic acid (TCA) cycle is the central hub of energy metabolism, macromolecular synthesis, and redox homeostasis. Multiple enzymes associated with the TCA cycle are mutated or imbalanced in cancer, leading to characteristic metabolic and epigenetic changes associated with disease transformation and progression [18]. Subsequent results of GSEA enrichment analysis of the high-risk group demonstrated its involvement in cellular energy metabolism, cell cycle regulation, and TGF-beta signaling pathway, which were tightly related to tumor progression [19–21]. GSEA enrichment analysis in the low-risk group was tightly associated with immune-related pathways. Similarly, poorer survival probabilities of the high-risk group were identified. The above consistently suggested the promotion of ferroptosis subcluster-related modular genes on growth, metastasis, and prognosis.

In addition, a risk-scoring model developed according to three ferroptosis subcluster-associated modular genes had excellent efficacy in independently assessing the OS prognosis at 1, 3, and 5 years in the training and testing data sets. We found that metastatic status and risk score were as well independent factors influencing the OS prognosis. Further integration of a nomogram with OS clinical features contributed to an optimal predictive ability for the OS survival rate. In this nomogram, risk score based on genetic features related to ferroptosis were the highest weighted scores, followed by metastatic status and tumor site. Finally, immunohistochemical experiments verified the protein expression of three ferroptosis subcluster-associated modular genes (*LRRC1*, *ACO2*, and *CTNNBIP1*), for which the model was constructed further validate the accuracy of our constructed risk-scoring model. These results have a crucial referential value regarding the clinical management and prognosis prediction for OS.

Our risk-scoring model consists of three ferroptosis subcluster-related modular genes whose value in tumors has been described in previous studies. LRRC1 was a LAP protein essential for controlling parietal basal cell polarity and proliferation [22]. Studies have demonstrated that increased LRRC1 expression promotes malignant biological behavior in hepatocellular carcinoma and cholangiocarcinoma tumor cells [23, 24]. ACO2 is a nuclear-encoded mitochondrial protein, and the decreased ACO2 was one independent predictive factor of poor prognosis for gastric cancer patients [25]. CTNNBIP1 is a *β*-linked protein interaction protein and could inhibit the binding of the *β*-linked protein to TCF, thus adversely regulating the Wnt/*β*-linked protein pathway [26]. CTNNBIP1 also negatively affects cancer progression. Downregulating CTNNBIP1 could enhance lung adenocarcinoma progression [27], while the upregulation suppressed glioma cell proliferation [28]. The risk-scoring model incorporating the above genes responds well to the prognostic status of patients.

Given the recent surprising effects and clinical importance of novel immunotherapies, including PD-1/PD-L1 blockade [29], our team then investigated the model predictability on the benefits of immunotherapy, followed by exploring the differential expression of the immune checkpoint-related PD-1 (PDCD1) and PD-L1 (CD274) genes. Both genes showed low expression in the high-risk subgroup, indicating insensitivity to therapy. And several immune checkpoint-related genes showed similar changes, such as B7-2 (CD86), B7-H3 (CD276), CD40, and CD40L (CD40LG). On the contrary, immune checkpoint-related genes of appeal were highly expressed in the low-risk group. These were consistent with the enrichment of immune-related BP in the low-risk group. The above indicated the insensitivity to tumor immunotherapy in patients of high risk.

Axitinib, an inhibitor of the receptor tyrosine kinase (including VEGF receptor [VEGFR] 1-3) [30], inhibits the VEGF/VEGFR signaling, disrupting its blood supply, and causing tumor cells to “starve”, thus exerting antitumor activity. Axitinib has been applied in treating patients with recurrent or refractory OS [31]. Cytarabine, a nucleoside analog, has been proved with activity against Ewing sarcoma [32]. Steckiewicz et al. found that Cytarabine induced cell death in OS cells [33]. Roscovitine is a purine analogue that competes with ATP for binding to cell cycle protein-dependent kinase (CDK). Roscovitine is a 2,6,9-trisubstituted purine analogue of olomoucine and competes with ATP for binding to cell cycle protein-dependent kinase (CDK) [34]. Vella et al. found that targeting CDK with Roscovitine increased OS cell sensitivity to DNA-damaging drugs [35]. We demonstrated that for Axitinib and Cytarabine, the IC50s were lower in the high-risk group, indicating a higher sensitivity to the targeted drug. In contrast, Roscovitine showed a greater IC50 in the high-risk group. The different sensitivity of two groups to three targeted drugs on appeal may lead to new ideas for individualized therapy of OS patients.

Meanwhile, some shortcomings existed in this study. Firstly, the number of samples obtained from GEO or TARGET databases in this study was limited. Further studies with larger samples are required to fully assess the efficacy of models and clarify potential mechanisms in the future. Second, due to the relative incompleteness of the data, the line graphs lack other important clinical features (e.g., clinical stage of osteosarcoma, and patient treatment information). In addition, specific cancer genes represented by RAS and TP53 may also impact patient prognosis [36, 37]. The expression of these cancer genes has not been subgroup analyzed and integrated into the column line graph in this study. Despite the excellent efficacy of the model for prognosis prediction, its effectiveness generally has room for further improvement, which will be a major area for future studies. Third, although this study has successfully validated the test cohort and verified the protein expression of the three modeled genes, many external validation studies are also required for accuracy verification. Finally, this study's conclusions on the relation of the risk-scoring model to immune checkpoint markers and response to targeted therapy lack further validation. Although we state its plausibility in the discussion section, the evidence remains weak, and additional confirmation by basic and clinical trials is needed. The different sensitivities of the high-risk and low-risk groups to the three targeted drugs involved in the current study deserve further investigation.

## 5. Conclusion

To sum up, two ferroptosis-associated subclusters in OS with different prognoses were identified. Then, a risk-scoring model, constructed according to three ferroptosis subcluster-related modular genes, showed good independent predictive power for the OS prognosis. In addition, the nomogram incorporating risk score and clinical characteristics showed outstanding advantages in predicting patient prognosis. The association of the risk-scoring model with immune checkpoint markers and the response to targeted therapy provides new ideas for targeted treatment of OS. Of course, more validation studies are needed in the future.

## Figures and Tables

**Figure 1:** Identification of ferroptosis subcluster. (a–c) Identification of subclusters based on the minimal crossover between cluster strata. (d) Survival analysis of two subclusters. CDF: cumulative distribution function; FRG: ferroptosis-related gene.

**Figure 2:** Consensus weighted gene coexpression network analysis and construction of the prognostic model. (a) The hierarchical clustering tree was obtained using the dynamic cutting method. (b) Pearson correlation matrix of the module features. (c) Forest map of ferroptosis subcluster-related modular genes associated with overall survival by Cox regression analysis. (d, e) Diagram of the optimal number of genes and coefficient spectrum in the LASSO regression model, respectively. (f) Forest map of three prognostic markers associated with overall survival by multivariate analysis.

**Figure 3:** Verification of the prognostic model in the training set. (a) Risk score plot. (b) Survival status scatters the plot. (c) Heat map for the expression of LRRC1, ACO2, and CTNNBIP1. (d) K-M curves. (e) Receiver operating characteristic (ROC) curves for overall survival. (f) Calibration curves plot.

**Figure 4:** Verification of the prognostic model in the testing set. (a) Risk score plot. (b) Survival status scatters the plot. (c) Heat map for the expression of LRRC1, ACO2, and CTNNBIP1. (d) K-M curves. (e) Receiver operating characteristic (ROC) curves for overall survival. (f) Calibration curves plot.

**Figure 5:** Relationships of model and clinical eigenvalues. (a, b) Forest plots of the Cox regression analysis of univariate and multivariate, respectively. (c) Box plots of the relationship between the model and clinical characteristics. Age: 0, older than 15 years old; 1, less than 15 years old. Gender: 0, male; 1, female. Tumor location: 0, lower extremity; 1, upper extremity. Metastases: 0, no metastasis; 1, metastasis at diagnosis; 2, metastasis after diagnosis.

**Figure 6:** Establishment of the nomogram. (a) Nomogram for overall survival prediction. Age: 0, older than 15 years old; 1, less than 15 years old. Gender: 0, male; 1, female. Tumor location: 0, lower extremity; 1, upper extremity. Metastases: 0, no metastasis; 1, metastasis at diagnosis; 2, metastasis after diagnosis. (b) MultiROC analyses for risk score and clinical characteristics. (c) Decision curve analysis (DCA) of the nomogram. The net benefit was plotted versus the threshold probability. m1, age; m2, gender; m3, tumor location; m4, metastases; m5, riskScore; m6, combine.

**Figure 7:** Functional enrichment analysis for the “turquoise” module. (a) Barplot and (b) Bubble plot of GO enrichment analysis. (c) Barplot and (d) Bubble plot of KEGG enrichment analysis.

**Figure 8:** Gene set enrichment analysis. (a, b) GO enrichment analyses for the high-risk and low-risk groups, respectively. (c, d) KEGG enrichment analyses for the high-risk and low-risk groups, respectively.

**Figure 9:** Association of the risk-scoring model with immune checkpoint markers and response to targeted therapies. (a) Expression of 20 immune checkpoint-related genes. (b–d) Prediction of response to targeted drugs.

**Figure 10:** qRT-PCR result of human osteoblast hFoB1 and human osteosarcoma cells U2-OS, MG-63.

**Figure 11:** Immunohistochemical staining of bone tissue in OS and paracancerous samples.

**Table 1:** Forward and reverse sequences of primers for LRRC1, CTNNBIP1, and ACO2.

Primer	Sequence (5′ to 3′)
LRRC1-F	AGACACAGACTACACCACAGGAGAG
LRRC1-R	CGCTCGTTCCAGGCTTCATCAG
CTNNBIP1-F	GAGGAGATGTACATTCAGCAGA
CTNNBIP1-R	GTTGACCACCCCTGCATAG
ACO2-F	TCAAGCTATGAAGATATGGGGC
ACO2-R	GATCCCTCAAGATCTGTGCATA
GAPDH-F	CAGGAGGCATTGCTGATGAT
GAPDH-R	GAAGGCTGGGGCTCATTT

## Data Availability

The data used to support the findings of this study are included in the article.

## Additional Points

*Manuscript Contribution to the Field.* The interaction of ferroptosis in OS development may provide new insights into exploring molecular mechanisms and targeted therapies for OS patients. However, more validation studies are needed in the future.
